# Intelligent Algorithm-Based Echocardiography to Evaluate the Effect of Lung Protective Ventilation Strategy on Cardiac Function and Hemodynamics in Patients Undergoing Laparoscopic Surgery

**DOI:** 10.1155/2022/9349027

**Published:** 2022-06-30

**Authors:** Huijuan Wang, Chao Gong, Yi Zhang, Yun Wang, Xiaoli Wang, Xiao Zhao, Lianhua Chen, Shitong Li

**Affiliations:** Department of Anesthesiology, Shanghai General Hospital of Nanjing Medical University, Shanghai 201600, China

## Abstract

The aim of this study was to analyze the effect of optimal pulmonary compliance titration of PEEP regimen on cardiac function and hemodynamics in patients undergoing laparoscopic surgery. 120 patients undergoing elective laparoscopic radical resection of colorectal cancer were included as the study subjects and randomly divided into the experimental group (*n* = 60) and the control group (*n* = 60). The control group had a fixed positive end-expiratory pressure (PEEP) = 5 cmH_2_O. The experimental group had transesophageal ultrasound monitoring through on an improved noise reduction algorithm (ONLM) based on nonlocal mean filtering (NLM) according to optimal pulmonary compliance titration of PEEP. There was significant difference in cerebral oxygen saturation and blood glucose level at T4-T6 between the experimental group and the control group (*P* < 0.05); the signal-to-noise ratio (SNR), figure of merit (FOM), and structural similarity (SSIM) of ONLM algorithm were significantly higher than those of NLM algorithm and Bayes Shrink denoising algorithm, and the differences were statistically significant (*P* < 0.05); there was significant difference in stroke volume (SV) and cardiac output (CO) at T4-T6 between the experimental group and the control group (*P* < 0.05); there was significant difference in pH, partial pressure of carbon dioxide (PCO_2_), and PO_2_ at T4-T6 between the experimental group and the control group (*P* < 0.05); pH was higher, and PCO_2_ and PO_2_ were lower in the experimental group. The results showed that transesophageal ultrasound based on the ONLM algorithm can accurately assess cardiac function and hemodynamics in patients undergoing laparoscopic surgery. In addition, optimal pulmonary compliance titration of PEEP could better maintain arterial acid-base balance during perioperative period and increase cerebral oxygen saturation and CO, but this strategy had no significant effect on hemodynamics.

## 1. Introduction

With the arrival of aging society, more and more elderly patients need surgery, and laparoscopic surgery is rapidly promoted in clinical practice because of its advantages of less trauma, rapid recovery, and mild postoperative pain, so laparoscopic surgery for elderly patients is also increasing in clinical practice [1]. Elderly patients have reduced pulmonary compliance and respiratory function. Laparoscopic surgery with CO_2_ pneumoperitoneum can increase intra-abdominal pressure, elevate diaphragm, and further reduce pulmonary compliance in elderly patients, leading to decreased ventilation function and increased arterial partial pressure of carbon dioxide (PCO_2_); high intra-abdominal pressure compresses the inferior vena cava, venous resistance increases, blood stasis in the lower limbs, venous return blood volume decreases, and left ventricular end diastolic volume decreases, resulting in decreased cardiac output (CO). The nervous system of elderly patients is also changed, and cerebral blood flow is also reduced by about 10%-20% in proportion to neural cell reduction. Many elderly patients have varying degrees of mental disorders and cognitive dysfunction after surgery. Postoperative cognitive dysfunction (POCD) has a serious impact on the high level of self-care needs and quality of life of elderly patients, so there are many clinical studies on the causes and mechanisms of POCD, which are still not fully understood. There are many studies that suggest that POCD in elderly patients is related to the decrease of cerebral oxygen saturation (rSO_2_) during operation in addition to age [2–5].

In recent years, lung protective ventilation strategy has been consistently advocated in clinical practice. Lung protective ventilation strategies, alone or in combination with low tidal volume, positive end-expiratory pressure (PEEP), and lung recruitment, have been shown to improve pulmonary oxygenation and lung physiology and reduce the occurrence of postoperative pulmonary complications in elderly patients [6]. However, different patients have different history of underlying diseases and are affected by surgical methods and pneumoperitoneum. Adjusting ventilation parameters based on experience alone is far from meeting clinical needs. At present, the controversy is more about the PEEP value, and when the PEEP setting is too low, the lung protection effect is weakened. When the PEEP setting is too high, it will not only cause lung injury but also further increase the intrathoracic pressure, block the venous return, reduce the return volume, and reduce the cardiac preload. Moreover, it can also increase alveolar pressure and pulmonary circulation resistance, affecting the right heart function and ultimately reducing CO. Some scholars believe that PEEP titration according to the optimal pulmonary dynamic compliance method can obtain ideal oxygenation, ventilation dead space ratio, and other pulmonary oxygenation indices [7–9]. However, circulation instability may occur. What is the reason for this circulation instability and whether it will affect CO? Does CO affect blood pressure, cerebral perfusion, and cerebral oxygen saturation? Previous studies have not directly revealed whether ventilation under optimal pulmonary dynamic compliance has an impact on CO and cerebral oxygen saturation in elderly patients undergoing laparoscopic surgery.

Echocardiography can identify cardiac structural lesions and cardiac function by displaying the structure and movement of the heart and blood vessels and measuring blood flow velocity. It is the most important and cost-effective examination for cardiovascular specialties; plays an important role in the diagnosis of cardiac valvular diseases, cardiomyopathy, congenital heart disease, cardiac tumors, and pericardial diseases; and has the advantages of low cost, no radiation, and strong availability [10–12]. However, echocardiography is susceptible to interference such as signal attenuation and speckle noise, and the initial image quality obtained is poor. Artificial intelligence, which uses computers and machines to imitate the problem-solving and decision-making capabilities of human thinking, has developed rapidly in recent years and has been widely used in the field of medical image processing. Artificial intelligence algorithm combined with medical imaging technology is a very hot topic at present, and the use of artificial intelligence algorithm to enhance the image and improve the quality of the image can better assist physicians in clinical evaluation [13, 14]. Based on this, it intends to use intelligent algorithm-based simultaneous monitoring of transesophageal echocardiography (TEE), cerebral oxygen saturation, and respiratory dynamics to observe and compare the CO and cerebral oxygen saturation of elderly patients undergoing laparoscopic surgery ventilated under two PEEP values (one PEEP = 5 cmH_2_O, one is based on optimal pulmonary compliance titration of PEEP) and analyze the relationship between cerebral oxygen saturation and CO. It is to provide a basis for more accurate individualized anesthesia management and better prognosis in elderly patients undergoing laparoscopic surgery.

## 2. Materials and Methods

### 2.1. Study Subjects

In this study, 120 patients (estimated operation time > 120 min) undergoing elective laparoscopic radical resection of colorectal cancer in hospital from October 2019 to January 2021 were selected as the study subjects. The patients were randomly divided into experimental group (*n* = 60) and control group (*n* = 60). The control group had fixed PEEP = 5 cmH_2_O. The experimental group was based on optimal pulmonary compliance titration of PEEP. This study was approved by ethics committee of hospital, and the patients and their families signed the informed consent form.

Inclusion criteria are as follows: American Society of Anesthesiologists (ASA) grades I-II, patients aged ≥ 65 years, patients without respiratory and circulatory system diseases, patients with normal liver and kidney function, patients with normal coagulation function, and patients with normal electrolytes.

Exclusion criteria are as follows: patients with anemia and malnutrition, patients with history of neurological diseases and mental illness, patients with absolute and relative contraindications to esophageal ultrasound, preoperative use of drugs that may affect hemodynamics and other unlicensed drugs, patients with failed esophageal ultrasound probe placement, intraoperative accidents (including hemodynamic disorders), and pregnant women.

### 2.2. Treatment Regimen

All patients were fasted for 8 hours before operation. After admission, the upper limb venous access was opened. 500-1,000 mL sodium lactate Ringer's solution was supplemented according to the preoperative loss. The monitor was connected. The electrocardiogram (ECG), upper limb noninvasive blood pressure (NIBP), and pulse oxygen saturation (SpO_2_) were routinely monitored. Left radial artery puncture (Allen test negative) and right internal jugular vein puncture were performed under local anesthesia with lidocaine. Left and right cerebral oxygen saturation was monitored as a basal value during air aspiration.

After 3 minutes of mask ventilation with air oxygen mixture > 6 L/min, 0.3-0.5 *μ*g/kg sufentanil, 1.5-2 mg/kg propofol, and 6-9 mg/kg rocuronium were used, endotracheal intubation was carried out, and mechanical ventilation was performed with a ventilator after successful intubation. The suction oxygen flow was 1 L/min, and the oxygen concentration was 60%. Respiratory parameters were adjusted: volume of tide (VT) according to ideal body weight, 9 mL/kg; respiratory rate (RR), 14 breaths/min; and inspiratory and expiratory ratio, 1 ∶ 1.5. Esophageal ultrasound was placed to monitor CO after the patient was inserted with an endotracheal tube. Lung protective ventilation strategy was implemented 10 min after the start of pneumoperitoneum, VT was adjusted to 6 mL/kg, and PEEP = 5 cmH_2_O was set after recruitment maneuver in fixation PEEP group; PEEP was titrated according to optimal lung compliance after recruitment in the titration PEEP group, and after optimal lung compliance was achieved, PEEP was fixed, and RR was adjusted according to end-tidal carbon dioxide partial pressure (35-45 mmHg) in both groups.

Intraoperative anesthesia is maintained by inhalation of desflurane (0.9–1.3 MAC), intermittent rapid injections of sufentanil and rocuronium, and rapid injections of vasoactive agents. After the end of surgery, 2 mg neostigmine and 1 mg atropine were intravenously injected for routine antagonism. After the patient was fully awake, the endotracheal tube was removed and sent to the resuscitation room.

### 2.3. Noise Reduction Algorithm Based on Nonlocal Mean Filtering (NLM)

The principle of NLM is to calculate the weighted sum of pixel values of all pixels in the rectangular window, and the weight follows Gaussian distribution. If the noise image is set as *p*, the pixel *x* of the image after noise reduction can be expressed as follows.

(1) $$\begin{array}{c} p=\left\{p\left(x\right)\left|x\in K\right.\right\}, \end{array}$$

(2) $$\begin{array}{c} p\left(x\right)*=\underset{y\in K}{\sum }\varphi \left(x,y\right)p\left(y\right), \end{array}$$

where *p*(*x*) represents the gray value of pixel *x* and *φ*(*x*, *y*) represents the weight, which is determined by the similarity of gray distribution in the field of pixel *x* and pixel *y*. Pixel *x* is set as the center, and setting the domain window of pixel *x* is set as *V*_*x*_; when reconstructing pixel *x*, the shared weight of another pixel *y* can be expressed as follows.

(3) $$\begin{array}{c} \varphi \left(x,y\right)=\frac{\exp-\left(Z\left(V_{x},V_{y}\right)/\alpha^{2}\right)}{A\left(x\right)}, \end{array}$$

where *Z*(*V*_*x*_, *V*_*y*_) represents the distance between two windows, *α* represents the change control parameter of weight, and *A*(*x*) represents the normalization parameter of weight, which is used to ensure ∑_*y*∈*K*_*φ*(*x*, *y*) = 1. Then, the *A*(*x*) can be expressed as follows:

(4) $$\begin{array}{c} A\left(x\right)=\underset{y\in K}{\sum }\exp-\frac{Z\left(V_{x},V_{y}\right)}{\alpha^{2}}. \end{array}$$

Gaussian weighted Euclidean distance was used to measure the distance between two windows.

(5) $$\begin{array}{c} Z\left(V_{x},V_{y}\right)={\left\|P\left(V_{x}\right)-P\left(V_{y}\right)\right\|}_{2,\eta }^{2}, \end{array}$$

where *η* means the standard deviation of the weighted Gaussian kernel, *P*(*V*_*x*_) represents the gray vector composed of the gray levels of all pixels in the domain window *V*_*x*_ of pixel *x*, and *P*(*V*_*x*_) = [*p*^1^(*x*), *p*^2^(*x*), *p*^3^(*x*),⋯,*p*^*m*^(*x*)]^*D*^ Equation (5) is substituted into Equation (2); the nonlocal mean filter can be obtained.

(6) $$\begin{array}{c} P\left(x\right)*=\frac{\sum_{y\in K}p\left(y\right)\exp-\left({\left\|P\left(V_{x}\right)-P\left(V_{y}\right)\right\|}_{2,\eta }^{2}/\alpha^{2}\right)}{\sum_{y\in K}\exp-\left({\left\|P\left(V_{x}\right)-P\left(V_{y}\right)\right\|}_{2,\eta }^{2}/\alpha^{2}\right)}. \end{array}$$

The nonlocal mean filter can denoise one pixel through all pixels in the image, but the calculation is cumbersome because the calculation is oriented to all pixels. Therefore, on the premise of ensuring the noise reduction effect, the processing range is reduced to a certain range centered on pixel *x* (*y* ∈ ℧_*x*_).

(7) $$\begin{array}{c} P\left(x\right)*=\frac{\sum_{y\in {℧}_{x}}p\left(y\right)\exp-\left({\left\|P\left(V_{x}\right)-P\left(V_{y}\right)\right\|}_{2,\eta }^{2}/\alpha^{2}\right)}{\sum_{y\in {℧}_{x}}\exp-\left({\left\|P\left(V_{x}\right)-P\left(V_{y}\right)\right\|}_{2,\eta }^{2}/\alpha^{2}\right)}. \end{array}$$

The above is the improved NLM algorithm, which is set as ONLM.

### 2.4. Noise Reduction Indexes

The traditional NLM algorithm [15] and Bayes Shrink denoising algorithm [16] are introduced to compare with the proposed ONLM algorithm.

Signal to noise ratio (SNR), figure of merit (FOM), and structural similarity (SSIM) are used as the noise reduction indexes of the algorithm.

The noise image is set as *f*(*x*) and the image after noise reduction as *g*(*x*).

SNR is the most direct way to evaluate the noise reduction effect of the algorithm, which can be expressed as follows.

(8) $$\begin{array}{c} \text{SNR}=10\log\left(\frac{\sum_{x\in K}\left(f^{2}\left(x\right)+g^{2}\left(x\right)\right)}{\sum_{x\in K}{\left(f\left(x\right)-g\left(x\right)\right)}^{2}}\right). \end{array}$$

SSIM can be used to display the structural similarity between denoised image and noisy image.

(9) $$\begin{array}{c} \text{SSIM}=\frac{\left(2\bar{f}\cdot \bar{g}+a_{1}\right)\left(2\eta_{fg}+a_{2}\right)}{\left({\bar{f}}^{2}\cdot {\bar{g}}^{2}+a_{1}\right)\left(\eta_{f}^{2}+\eta_{g}^{2}+a_{2}\right)},\\ a_{1}=0.013\left|\Pi \right|,\\ a_{2}=0.025\left|\Pi \right|, \end{array}$$

where *Π* represents the gray range of the image.

FOM can be used to evaluate image edge information.

(10) $$\begin{array}{c} \text{FOM}=\frac{\sum_{i=1}^{m_{l}}\left(1/\left(1+{cl}_{i}^{2}\right)\right)}{\max\left(m_{f},m_{g}\right)}, \end{array}$$

where *m*_*f*_ means the number of edge pixels of the noisy image, *m*_*g*_ represents the number of edge pixels of the denoised image, *l*_*i*_ indicates the minimum Euclidean distance between the edges of two images, and *c* is a constant.

### 2.5. Observation Indicators

Intraoperative general conditions are as follows: surgical name, surgical position, anesthesia time, analgesic dosage, operation time, blood loss, blood transfusion volume, infusion volume, intraoperative application of vasoactive drugs, ICU admission time, and total hospital stay.

Observation indicators are as below: before induction of anesthesia (T0), 5 minutes after successful intubation (T1), 10 minutes after pneumoperitoneum (T2); 10 minutes after satisfactory PEEP adjustment (T3); 30 minutes after satisfactory PEEP ventilation (T4); 60 minutes after satisfactory PEEP ventilation (T5); no pneumoperitoneum after laparotomy (T6). Heart rate (HR), systolic blood pressure (SBP), diastolic blood pressure (DBP), mean arterial pressure (MAP), pulse oxygen saturation (SpO_2_), body temperature, blood glucose, cerebral oxygen saturation (rSO_2_), blood flow velocity time integral (VTI), stroke volume (SV), CO, and arteriovenous blood gas analysis (pH, PO_2_, PCO_2_) were recorded.

### 2.6. Statistical Methods

Data processing was analyzed by the SPSS 19.0 statistical software, measurement data were expressed as mean ± standard deviation ($\overset{¯}{\text{x}}\pm s$), and enumeration data were expressed as percentage (%). One-way analysis of variance was used for pairwise comparisons. The difference was statistically significant at *P* < 0.05.

## 3. Results

### 3.1. Comparison Results of Noise Reduction Performance of Algorithms

The noise reduction indicators SNR, FOM, and SSIM of the images by the ONLM algorithm were significantly higher than those by the NLM algorithm and the Bayes Shrink denoising algorithm, and the differences were statistically significant (*P* < 0.05) (Figure 1).

Figure 2 shows the noise reduction effect of the three algorithms on echocardiography. Compared with the original image, the three algorithms had obvious effects on the noise reduction processing of echocardiography, in which the image after noise reduction by NLM algorithm had a certain improvement in brightness and sharpness, but the overall background was relatively dim, and there was no significant difference in detail comparison; the image after noise reduction by Bayes Shrink denoising algorithm also had a significant improvement in sharpness and brightness, but there was an overexposure problem, which affected the tissue detail display; the overall quality of the image after noise reduction by ONLM algorithm was the highest, the noise and pseudo were greatly reduced, and there was a better sharpness and brightness.

### 3.2. Comparison of General Data

There were no significant differences in gender, age, height, weight, marital status, education level, diabetes, hypertension, smoking, alcohol consumption, and ASA classification between the experimental group and the control group (*P* > 0.05) (Figure 3).

### 3.3. Comparison of Intraoperative General Conditions

There was no significant difference in anesthesia time, operation time, pneumoperitoneum time, infusion volume, blood loss, urine volume, ICU stay, and hospital stay between the experimental group and the control group (*P* > 0.05) (Figure 4).

### 3.4. Comparison of Hemodynamic Parameters

There was no significant difference in HR, SBP, DBP, MAP, and SpO_2_ at T1-T6 between the experimental group and the control group (*P* > 0.05) (Figure 5).

### 3.5. Comparison of Cerebral Oxygen Saturation, Body Temperature, and Blood Glucose Level

There was no significant difference in the body temperature at T1-T6 between the experimental group and the control group (*P* > 0.05); there was no significant difference in the cerebral oxygen saturation and blood glucose level at T1-T3 between the experimental group and the control group (*P* > 0.05); there was significant difference in the cerebral oxygen saturation and blood glucose level at T4-T6 between the experimental group and the control group (*P* < 0.05) (Figure 6).

### 3.6. Comparison of Cardiac Function Indexes

There was no significant difference in the VTI at T1-T6 between the experimental group and the control group (*P* > 0.05); there was no significant difference in the SV and CO at T1-T3 between the experimental group and the control group (*P* > 0.05); there was significant difference in the SV and CO at T4-T6 between the experimental group and the control group (*P* < 0.05) (Figure 7).

### 3.7. Comparison of Arteriovenous Blood Gas Analysis Indicators

There was no significant difference in pH, PCO_2_, and PO_2_ at T1-T3 between the experimental group and the control group (*P* > 0.05); there was significant difference in pH, PCO_2_, and PO_2_ at T4-T6 between the experimental group and the control group (*P* < 0.05); pH was higher, and PCO_2_ and PO_2_ were lower in the experimental group (Figure 8).

## 4. Discussion

Laparoscopic surgery is a minimally invasive method developed in recent years and a development trend of clinical surgical treatment, with the advantages of less trauma to patients, less intraoperative bleeding, and beautiful wounds [17, 18]. Of course, laparoscopic surgery also has obvious disadvantages, such as pneumoperitoneum during surgery will lead to acidosis, subcutaneous emphysema, and respiratory dysfunction, so how to perform lung protective ventilation in laparoscopic surgery has been a key topic for scholars [19–22]. Based on this, 120 patients undergoing elective laparoscopic radical resection of colorectal cancer were included as the study subjects and randomly divided into the experimental group (*n* = 60) and the control group (*n* = 60). The control group had a fixed PEEP = 5 cmH_2_O. The experimental group underwent transesophageal ultrasound monitoring according to the optimal pulmonary compliance titration of PEEP. In order to better perform imaging evaluation, an improved noise reduction algorithm ONLM based on NLM was also proposed and compared with the traditional NLM algorithm and Bayes Shrink algorithm, and the results showed that the noise reduction indicators SNR, FOM, and SSIM of the image by the ONLM algorithm were significantly higher than those by the NLM algorithm and Bayes Shrink denoising algorithm, and the difference was statistically significant (*P* < 0.05), which suggested that the proposed ONLM algorithm was superior to the NLM algorithm and Bayes Shrink denoising algorithm for the noise reduction performance of the original image and can better improve the image quality. From the image display of noise reduction by the three algorithms, the overall quality of the image after noise reduction by the ONLM algorithm was the highest, the noise and artifact were greatly reduced, and there was better clarity and brightness, which corresponded to the above quantitative data results.

Comparison of hemodynamic parameters between the two groups showed that there was no significant difference in HR, SBP, DBP, MAP, and SpO_2_ at T1-T6 between the experimental group and the control group (*P* > 0.05), indicating that optimal pulmonary compliance titration of PEEP had no significant effect on hemodynamics in patients undergoing laparoscopic surgery [23]. The cerebral oxygen saturation and blood glucose level at T4-T6 in the experimental group were significantly different from those in the control group (*P* < 0.05). Cerebral oxygen saturation can indicate the balance between cerebral oxygen supply and demand, and the imbalance between cerebral oxygen supply and demand may trigger cerebral ischemia and hypoxia, increase the incidence of complications, and affect the prognosis of patients, so it is very important to maintain the appropriate balance between cerebral oxygen supply and demand in patients [24, 25]. The results indicated that compared with fixed PEEP = 5 cmH_2_O, optimal pulmonary compliance titration of PEEP could better maintain cerebral oxygen supply and demand balance and blood glucose level and reduce the prognostic risk. SV refers to the volume of blood ejected from one ventricle in one heartbeat. CO is an important index to evaluate the efficiency of circulatory system. CO is largely commensurate with the metabolic rate of systemic tissue cells. Comparison of cardiac function indicators showed that there were significant differences in SV and CO at T4-T6 between the experimental group and the control group (*P* < 0.05). This is similar to the study results of Luecke and Pelosi [26], indicating that optimal pulmonary compliance titration of PEEP can effectively maintain SV and CO in patients undergoing laparoscopic surgery and avoid cardiac function damage caused by surgery. pH, PCO_2_, and PO_2_ at T4-T6 in the experimental group were significantly different from those in the control group (*P* < 0.05), and pH was higher, and PCO_2_ and PO_2_ were lower in the experimental group, which indicated that optimal pulmonary compliance titration of PEEP could better maintain arterial acid-base balance and avoid the occurrence of acidosis. To sum up, the ONLM algorithm proposed in this work showed a good effect on ultrasonic image processing and a high clinical promotion value. In addition, optimal lung compliance titration of PEEP can effectively maintain the acid-base balance of arterial blood in patients during the perioperative period and avoid problems such as cerebral oxygen supply and demand imbalance, acidosis, and cardiac function damage caused by surgery. However, this strategy had no significant effect on hemodynamics.

## 5. Conclusion

The results showed that the ONLM algorithm is superior to the NLM algorithm and Bayes Shrink denoising algorithm for the new noise reduction performance of ultrasound, which can better improve the image quality. Optimal pulmonary compliance titration of PEEP can better maintain arterial acid-base balance and increase cerebral oxygen saturation and CO in patients to avoid the imbalance of cerebral oxygen supply and demand, acidosis, cardiac function damage, and other problems caused by surgery, but this strategy has no significant effect on hemodynamics. In conclusion, it provides a theoretical reference for the selection of lung-protective ventilation regimen in patients undergoing clinical laparoscopic surgery. However, the included samples were from the same hospital, which may affect the generalizability of the results. Moreover, there was no follow-up after discharge. There was no long-term prognosis data of the patients. The samples will be further included for more in-depth discussion.

## Figures and Tables

**Figure 1:** Comparison of noise reduction indexes of three algorithms: (a) SNR; (b) FOM; (c) SSIM. ^∗^Compared with ONLM algorithm, *P* < 0.05.

**Figure 2:** Demonstration of the noise reduction effect of three algorithms on echocardiography: (a) the original image; (b) the NLM algorithm; (c) the Bayes Shrink denoising algorithm; (d) the ONLM algorithm.

**Figure 3:** Comparison of general data between the experimental group and the control group: (a) gender; (b) age, height, and weight; (c) marital status; (d) education level; (e) diabetes, hypertension, smoking, and alcohol consumption; (f) ASA classification.

**Figure 4:** Comparison of intraoperative general conditions between the experimental group and the control group: (a) anesthesia time, operation time, and pneumoperitoneum time; (b) infusion volume; (c) blood loss and urine volume; (d) ICU stay and hospital stay.

**Figure 5:** Comparison of hemodynamic parameters between the experimental group and the control group: (a–e) HR, SBP, DBP, MAP, and SpO_2_, respectively.

**Figure 6:** Comparison of cerebral oxygen saturation, body temperature, and blood glucose level between the experimental group and the control group: (a–c) cerebral oxygen saturation, body temperature, and blood glucose level, respectively. ^∗^Compared with the experimental group, *P* < 0.05.

**Figure 7:** Comparison of cardiac function indexes between the experimental group and the control group: (a–c) blood flow VTI, SV, and CO, respectively. ^∗^Compared with the experimental group, *P* < 0.05.

**Figure 8:** Comparison of arteriovenous blood gas analysis indicators between the experimental group and the control group: (a–c) pH, PCO_2_, and PO_2_, respectively. ^∗^Compared with the experimental group, *P* < 0.05.

## Data Availability

The data used to support the findings of this study are available from the corresponding author upon request.
